# Low Testosterone Level and Risk of Adverse Clinical Events among Male Patients with Chronic Kidney Disease: A Systematic Review and Meta-Analysis of Cohort Studies

**DOI:** 10.1155/2022/3630429

**Published:** 2022-09-10

**Authors:** Li Li, Huixiang Ju, Hao Jin, Hongmei Chen, Mingzhong Sun, Zhongwei Zhou

**Affiliations:** ^1^Department of Clinical Laboratory, Binhai County People's Hospital, Binhai, Yancheng, Jiangsu 224500, China; ^2^Department of Clinical Laboratory,Yancheng Third People's Hospital (The Yancheng School of Clinical Medicine of Nanjing Medical University, The Sixth Affiliated Hospital of Nantong University, The Affiliated Yancheng Hospital of Southeast University Medical College), Yancheng, Jiangsu 224001, China; ^3^Department of Blood Transfusion,Yancheng Third People's Hospital (The Yancheng School of Clinical Medicine of Nanjing Medical University, The Sixth Affiliated Hospital of Nantong University, The Affiliated Yancheng Hospital of Southeast University Medical College), Yancheng, Jiangsu 224001, China

## Abstract

The phenomenon of low testosterone level is extremely common in male patients with chronic kidney diseases (CKDs). This meta-analysis aimed to evaluate whether the low circulating testosterone could independently predict adverse outcomes among male patients with chronic kidney diseases (CKDs). The data till May 2022 were systematically searched from Pubmed, Web of Science, and Embase from inception. Studies meeting the PICOS (population, intervention/exposure, control/comparison, outcomes, and study design) principles were included in this meta-analysis. Study-specific effect estimates were pooled using fixed-effects (*I*^2^ > 50%) or random-effects models (*I*^2^ < 50%). Ultimately, 9 cohort studies covering 5331 patients with CKDs were involved in this meta-analysis. The results suggested that per 1-standard deviation (SD) decrease in total testosterone independently increased the risk of all-cause mortality by 27% [hazard risk (HR) 1.27, 95% confidence interval (CI) 1.16–1.38], cardiovascular mortality by 100% (HR 2.00, 95% CI 1.39–2.86), cardiovascular events by 20% (HR 1.20, 95% CI 1.04–1.39), and infectious events by 41% (HR 1.41, 95% CI 1.08–1.84). Besides, with per 1-SD decrease in free testosterone, the risk of overall adverse events increased by 66% (HR 1.66, 95% CI 1.34–2.05). Stratified analyses indicated that the negative relationship of the total testosterone with all-cause death risk was independent of factors involving age, race, body mass index, diabetes, hypertension, C-reactive protein, creatinine, and sex hormone binding globulin. In conclusion, it was identified that low endogenous testosterone could serve as an independent predictor of adverse clinical events among male patients with CKDs.

## 1. Introduction

Chronic kidney diseases (CKDs) may signify a high risk of adverse clinical events, which affect approximately 10% of the world population [1]. Epidemiological studies have demonstrated that the incidence of CKDs is higher among women than age-matched men, while male patients show a faster development to end-stage renal diseases (ESRDs) [2, 3]. On the other hand, postmenopausal women display a higher rate of CKDs in comparison to premenopausal females, accompanied with a more rapid progression [4, 5]. These facts suggest that sex hormones may play a significant role in the development and progression of CKDs.

Testosterone as one of the primary male sex hormones is not only responsible for the regulation of reproductive function, but also involved in numerous physiological processes [6]. In healthy adult males, the level of endogenous testosterone exhibits a progressive decrease with age, especially in those aged over 40 years [7]. In pathological conditions such as metabolic abnormalities and inflammatory diseases, the decreased testosterone concentration would be more pronounced [8]. In a recent cross-sectional study covering 1222 men aged 40–70 years, endogenous testosterone deficiencies (total testosterone ≤3.46 ng/mL or free testosterone ≤72 pg/mL) were detected in more than half of the subjects; however, up to 97.2% of them, presented one or more comorbidities such as dyslipidemia, hypertension, and diabetes mellitus [9]. This distinction in the testosterone level from a physiologically moderate decrease with advancing age and pathologically significant reductions due to diseases may serve to predict the risk of adverse clinical events in certain conditions, such as CKDs.

Manipulated by the excretion, synthesis and degradation of various hormones, the kidney plays a vital role in maintaining body homeostasis [10, 11]. Therefore, patients with CKDs typically present varying degrees of hormone disorders. Previous studies have demonstrated a decreased level of endogenous testosterone in male suffering from CKDs, which held prognostic value in predicting adverse outcomes [12, 13], while these findings have failed to reach a consistence. Moreover, most of the findings were based on relatively small sample sizes. In this study, we systematically evaluated the prognostic significance of the low testosterone level in predicting the risk of adverse clinical events among male patients with CKDs based on a pooled analysis.

## 2. Methods

This systematic review was conducted following PRISMA guidelines [14], with the review protocol prospectively registered on INPLASY (registration number: INPLASY 202250085).

### 2.1. Search Strategy

The data from inception until May 1, 2022 were systematically searched PubMed, Web of Science, and EMBASE. The search strategies covered the following medical subject headings and free words: (“testosterone” OR “androgen”) AND (“chronic kidney disease,” “chronic renal failure,” “end-stage renal disease,” “ESRD,” “hemodialysis,” “peritoneal dialysis” OR “dialysis”) AND (“cohort,” “prospective,” “retrospective,” “longitudinal” OR “follow-up”). Reference lists of selected literature were also checked for additional studies.

### 2.2. Selection Criteria

Studies were included according to the following PICOS criteria: Population: patients with CKDs regardless of dialysis. Exposure: low circulating testosterone as risk factor. Comparators: lowest quantile vs. highest quantile or per unit/standard deviation (SD) change. Outcomes: adverse clinical events, such as cardiovascular events and mortality. Study design: cohort studies irrespective of prospective or retrospective designs. The exclusion criteria were as follows: (1) studies that reported an unadjusted hazard ratio (HR) and 95% confidence interval (CI), (2) follow-up period less than 1 year, (3) nonenglish language publications, (4) reviews, conference abstracts, editorials, case reports, intervention studies, or nonhuman studies.

### 2.3. Data Extraction and Quality Assessment

The study selection, data extraction, and quality assessment were independently conducted by two investigators, respectively, in which any disagreement was resolved by consensus or consulting a third author. For each involved study, the data of first author's name, the year of publication, study site, study design, patient type, sample size, age of patient, testosterone comparison, event number, multivariable-adjusted HR (95% CI), follow-up time and adjusted confounders were extracted. The methodological quality of the cohort studies included was evaluated using the Newcastle-Ottawa Scale (NOS) [15], which contained three domains and nine items, namely population selection, comparability, and outcome. The score ranged from 0 to 9 points, and studies scoring 7–9, 4–6, and 0–3 were considered to be of a high, moderate, and low quality, respectively.

### 2.4. Statistical Analysis

Statistical analyses were carried out using Stata (version 15.0; Stata Corp LP, College Station, TX). Among the 9 studies included, the effect estimates were reported to predict adverse outcomes based on various categories (e.g., dichotomous categories, tertiles, or quintiles) in exposure. For a consistent and quantifiable comparison, the effect estimates were transformed to per 1-standard deviation (SD) decrease of testosterone concentration according to the previously established methods [16]. For the implementation, the circulating testosterone concentration was assumed to follow a lognormal distribution, with a linear relationship existing between testosterone and the risk of adverse events in the log scale. On this basis, the adjusted effect estimates for the lowest and the highest tertile of testosterone level corresponded to 2.18 SD units. In terms of dichotomous categories (low vs. high) and quintile groups (bottom vs. top), the scaling factors were 1.59 and 2.80, respectively. For 1 study [17] in which per 1-unit changes were reported, the estimates were directly converted into HR (95% CI) associated with per 1-SD decrease in testosterone. Heterogeneity was evaluated using *I*^2^ statistics, with an *I*^2^ value of >50% considered significantly heterogeneous. If the heterogeneity was not significant, a fixed-effects model was utilized to pool data; otherwise, a random-effects model would be chosen. Subgroup analyses were conducted to obtain more detailed information. Sensitivity analyses excluding 1 study at a time were carried out to investigate whether the results and the pooled effect estimates were driven by a single study. The potential publication biases were also assessed by inspecting funnel plots through the Egger's test.

A *P* value < 0.05 was deemed statistically significant.

## 3. Results

### 3.1. Literature Search

461 relevant studies were initially identified from the selected databases, remaining 226 records were identified after removing duplicates. According to the title and abstract review, 207 publications were excluded and 19 full-text articles were comprehensively evaluated. Ten studies were additionally excluded due to the lack of outcomes of interest. Finally, 9 studies [17–25] considered eligible were included in this meta-analysis (Figure 1).

### 3.2. Characteristics of Selected Studies

The baseline characteristics of the 9 included studies are summarized in Table 1, which were published from 2009 to 2018, totally covering 5331 patients treated with dialysis or nondialysis. Among these, 2 studies were from America, 2 from Turkey, and the other 5 from Sweden, Greece, Canada, Japan, and Taiwan, respectively. Patients treated with hemodialysis were enrolled in 6 studies, 2 of which only included patients with nondialysis CKDs, while 1 involved both hemodialysis and peritoneal dialysis patients. The sample size ranged from 111 to 2149, with the mean age from 52.0 to 71.7 years. The median follow-up time of studies included was from 1.2 to 5.0 years. According to the NOS scale, 4 studies were ranked as high quality and 5 as moderate quality.

### 3.3. Association between Total Testosterone (Per 1-SD Decrease) and Risk of Adverse Clinical Events

The relationship between the total testosterone and several adverse events were assessed covering all-cause deaths (8 studies), cardiovascular deaths (3 studies), cardiovascular events (3 studies), and infectious events (1 study). As depicted in Figure 2, per 1-SD decrease in the total testosterone corresponded to a higher risk of all-cause mortality (HR 1.27, 95% CI 1.16–1.38, *P* < 0.001), cardiovascular mortality (HR 2.00, 95% CI 1.39–2.86, *P* < 0.001), cardiovascular events (HR 1.20, 95% CI 1.04–1.39, *P* < 0.016), and infectious events (HR 1.41, 95% CI 1.08–1.84, *P* < 0.011). A random-effects model was used to conduct the pooled analysis of infectious events due to only 1 study (*I*^2^ = 100%), and the fixed-effects models were used for the other analyses considering the insignificant heterogeneity (*I*^2^ < 50%).

### 3.4. Association  between Free Testosterone (Per 1-SD Decrease) and Risk of Adverse Clinical Events

Three data points from 2 studies were included in the pooled analysis of the association between free testosterone and the risk of adverse clinical events [17, 20], since both all-cause and cardiovascular deaths were reported by Kyriazis et al. [20]. Given that each event was involved in 1 study only, we did not separately analyze these events, but did the effect estimates from all the adverse events. As presented in Figure 3, the risk of adverse clinical events increased by 66% (HR 1.66, 95% CI 1.34–2.05, *P* < 0.001) corresponding to per 1-SD decrease in free testosterone. No statistical heterogeneity was found in the pooled estimate (*I*^2^ = 0.0%), and the fixed-effects model was adopted.

### 3.5. Subgroup Analysis

Due to the small number of studies addressing other events, only subgroup analyses were carried out for the association between the total testosterone and all-cause mortality. The chosen studies were stratified according to the factors of study design, location, patient types, age, follow-up duration, and adjustment for race, body mass index (BMI), hypertension, diabetes, creatinine, C-reactive protein (CRP) as well as sex hormone binding globulin (SHBG). As indicated in Figure 4, except for the subgroup of patients with nondialysis CKDs (HR 1.13, 95% CI 0.99–1.28, *P*=0.062), all other subgroups displayed consistent findings with the overall results.

### 3.6. Sensitivity Analysis and Publication Bias

Similarly, a sensitivity analysis and publication bias were performed focused only on the relationship between the total testosterone and all-cause deaths. The leave-one-out sensitivity analysis indicated that no single study had significant effect on the overall effect estimate (Figure 5). However, an asymmetric shape was presented in a visual inspection of the funnel plot (Figure 6). The value of Egger's test (*P*=0.010) also suggested a possible publication bias.

## 4. Discussion

In the present meta-analyses, we evaluated the prognostic value of endogenous testosterone in predicting adverse clinical events among male patients with CKDs. The analyses suggested that per 1-SD decrease in total testosterone independently corresponded to the increased risk of all-cause deaths by 27%, cardiovascular deaths by 100%, cardiovascular events by 20%, and infectious events by 41%, accompanied with a significant relationship observed between free testosterone and the overall adverse events. The findings demonstrated that low endogenous testosterone could serve as an independent poor-prognostic factor for male individuals with CKDs.

Most recently, a meta-analysis conducted by Van der Burgh et al. [26] also indicated that a low testosterone level was associated with a higher risk of all-cause deaths and cardiovascular events. However, in their study, the pooled analysis was carried out based on continuous variables, dichotomous, and tertile groups, respectively, meaning that only 3 studies were involved in the conclusion that low testosterone might increase all-cause mortality risk (HR 1.98, 95% CI 1.36–2.89), in which effect estimates were reported based on dichotomous categories, while failing to obtain the significant relationship by pooling 2 studies where risk estimates were given based on extreme thirds. By contrast, our meta-analysis covered more studies (9 vs. 6). More significantly, an established approach was used [16] to convert various types of effect estimates into per SD changes of the testosterone level, through which we could have pooled more studies in a consistent manner in evaluating the prognostic value of circulating testosterone so as to acquire more convincing conclusions.

In the past few years, several meta-analyses have also evaluated the association between low endogenous testosterone and adverse outcomes in healthy and/or diseased populations. A recent meta-analysis indicated no association of the low endogenous testosterone with all-cause or cardiovascular deaths among community-dwelling men [27]. Another meta-analysis showed no significant relationship between low testosterone and the risk of cardiovascular diseases among healthy middle-aged men, but only a weak correlation observed among elderly men [28]. Yet, results of one meta-analysis involving a mixed population of healthy and unhealthy men revealed that low testosterone showed a significant predictive value for poor prognosis [29]. Therefore, male subjects' age and health status might affect the prognostic significance of low testosterone, and in light of this, testosterone replacement therapy (TRT) is considered to potentially reduce the risk of adverse events for diseased individuals and/or the elderly with a decreased level of testosterone, which, however, was suggested to increase the risk of cardiovascular-related events in a previous meta-analysis based on 27 placebo-controlled randomized trials with 2,994 male subjects [30]. For several decades, adverse cardiovascular events have not been reported in young men who received TRT due to testosterone deficiency elicited by organic diseases, including hypothalamic involvement, pituitary lesions, and testicular disease [31]. But for older men, or those with chronic diseases, such as diabetes and certain inflammatory diseases, whose low testosterone levels are induced by nonorganic diseases, whether TRT will contribute to an increased risk of major adverse events still remains controversial [32]. Most recently, Hudson et al. performed an updated meta-analysis covering 35 primary studies with 5601 participants, summarizing that TRT did not increase short- to medium-term cardiovascular risk in men with testosterone deficiency [33]. Hudson et al. also proposed that due to the lack of relevant data, the long-term safety of TRT remained to be proven. Indeed, TRT in the clinical application requires to be further evaluated. But anyway, a low level of circulating testosterone can serve as a useful biomarker for assessing the risk of adverse events, without the demand to know whether its decline is a cause or a consequence of some diseases, such as CKDs.

Of course, TRT has also been demonstrated to play a beneficial role in various aspects. For example, TRT has the potential to enhance the sexual health function, muscle strength, leg power, stair climbing power, and the anemia associated with chronic disease in older men [34, 35]. In addition, TRT has also been validated to be capable of alleviating insulin resistance and regulating glycolipid metabolism in hypogonadal men with type 2 diabetes mellitus or metabolic syndrome [36]. A newly published study reported that a 3-month-long TRT significantly improved the quality of life of male patients with moderate-to-severe CKDs, including hypogonadal symptoms, mental and physical function [37]. However, the current studies to evaluate the effects of TRT on clinical outcomes of CKDs are extremely lacked, and more randomized controlled trials can be expected in future.

The low circulating concentration of testosterone presented in patients with CKDs could be induced by several reasons. To begin with, a variety of hormones are metabolized and excreted in the kidneys [10, 11], in which the diseased kidneys result in abnormal hormone regulations, even leading to a disruption of the hypothalamic-pituitary-gonadal axis [38]. Next, diabetes, hypertension and atherosclerosis are common comorbidities found in patients with CKDs, of which the cumulative effect leads to a further reduction in their testosterone level [39]. Finally, CKDs are diseases of inflammation with a negative correlation with circulating testosterone and gradually enhanced as CKDs progress [40]. Although patients with CKDs presented the reduced testosterone levels in different degrees, it still remains unclear whether such reduction is a cause or consequence as previously mentioned. And it may act as a cause that few randomized controlled trials were conducted to evaluate the effect of TRT intervention on CKDs. One study involved in our meta-analysis showed no association of TRT with an increased mortality risk [21].

In our subgroup analysis, it was found that whether adjustment for diabetes, hypertension, or CRP did not exert distinct effect on the pooled effect estimates. Similarly, stratifications by adjustment of race, BMI, creatinine and SHBG also brought no different results. Since in all the studies included with age adjusted, the prognostic significance of circulating testosterone might be independent of race, BMI, age, hypertension, diabetes, creatinine, CRP, and SHBG. In addition, the differences in study designs, study sites, age strata, and follow-up durations did not produce inconsistence in estimation with the overall results. Only 1 study involving patients with nondialysis CKDs with stratification by patient types was of borderline significance (*P*=0.062). These results further suggested the independent prognostic significance of circulating testosterone for adverse events among patients with CKDs.

Our work has the following advantages. Our meta-analysis only covered studies with multivariable-adjusted effect estimates, which contributed to minimize the interference of the confounding factors on the prognostic significance of circulating testosterone. In addition, our pooled results were robust to a certain degree considering the insignificant heterogeneity between-studies. Several potential limitations should also to be mentioned. First of all, since only 3 data points from 2 studies were included in the meta-analysis evaluating the prognostic value of free testosterone, the analysis pointed to overall adverse events rather than the respective single events, which might lead to a confounding bias. Additionally, the limited number of studies included in this analysis might result in less convincing conclusion. Similar limitations should also be taken into account in evaluating the total testosterone for predicting cardiovascular deaths, cardiovascular events, and infectious events. Secondly, to facilitate a consistent comparative analysis, the effect estimates were converted into per SD changes of circulating testosterone level in the included studies. Despite as another major strength of our study, this conversion could also be a limitation, as it might introduce a degree of bias. Finally, the asymmetric funnel plot suggested the presence of potential publication biases. A possible explanation is that only studies in English and full texts were included, but not conference abstracts or nonenglish articles, which might result in a selection bias of our pooled analysis.

## 5. Conclusion

The present meta-analysis demonstrated that both total and free testosterone of a low level could serve as an independent prognostic factor of adverse clinical events for male patients with CKDs. Among them, the total testosterone was independently associated with a higher risk of all-cause deaths, cardiovascular deaths, cardiovascular events, and infectious events. Larger cohort studies are warranted to validate our findings in the future.

## Figures and Tables

**Figure 1:** The flow chart of the study selection process.

**Figure 2:** Forest plot of the association between per 1-SD decrease in total testosterone and adverse clinical events, including all-cause mortality, cardiovascular mortality, cardiovascular events, and infectious events. HR, hazard risk; CI, confidence interval.

**Figure 3:** Forest plot of the association between per 1-SD decrease in free testosterone and the overall adverse events. HR, hazard risk; CI, confidence interval.

**Figure 4:** Forest plot presenting subgroup analysis of the association between total testosterone and all-cause mortality. HR, hazard risk; CI, confidence interval.

**Figure 5:** Sensitivity analysis of the association between total testosterone and all-cause mortality. CI, confidence interval.

**Figure 6:** Funnel plot assessing potential publication bias for the association between total testosterone and all-cause mortality. HR, hazard risk.

**Table 1:** Summary of clinical studies included in meta-analysis.

Author/year	Region	Study design	Patient types	Sample size	Age (years)	Comparison	Event number/adjusted HR (95% CI)	Follow-up (years)	Adjusted confounders	Overall NOS
Carrero et al. 2011 [17]	Turkey	Prospective cohort	Nondialysis CKD	239	52.0 ± 12.0	Per unit increase	CV events: 72; total testosterone: 0.83 (0.78–0.88); free testosterone: 0.65 (0.53–0.80)	2.58	Age, eGFR, diabetes, CVD, CRP, albumin, FMD	5

Gungor et al. 2009 [18]	Sweden	Prospective cohort	HD	126	63.0 ± 17.8	Low vs. high	Total death: 65; 1.51 (0.86–2.72); CV death: 38; 2.00 (0.80–4.95)	3.42	Age, SHBG, diabetes, CVD, ACEI/ARB medication, IL-6, albumin, creatinine	5

Yilmaz et al. 2010 [19]	Turkey	Prospective cohort	HD	420	54 ± 13	Lowest tertile 3 vs. highest	Total death: 104; 1.49 (0.83–2.66)	2.67	Age, BMI, HD duration, diabetes, CVD, albumin, creatinine, CRP	7

Kyriazis et al. 2011 [20]	Greece	Prospective cohort	HD	111	65 ± 12	Low vs. high	Total death: 49; total testosterone: 2.81 (1.23–6.38); free testosterone: 2.62 (1.27–5.44); CV death: 28; total testosterone: 2.29 (0.78–6.72); free testosterone: 2.47 (0.92–6.64)	3.08	Age, BMI, CVD, HD vintage, CRP, albumin, PWV	6

Khurana et al. 2014 [21]	America	Retrospective cohort	Nondialysis CKD	2149	67.3 ± 11.3	Lowest quintile 5 vs. highest	Total death: 357; 1.420 (0.995–2.020)	2.3	Age, BMI, race, smoking, eGFR, cerebrovascular disease, diabetes, hypertension, CAD, CHF, hyperlipidemia, albumin, malignancy, testosterone medication	8

Bello et al. 2014 [22]	Canada	Prospective cohort	HD	623	60.7 ± 15.2	Lowest tertile 3 vs. highest	Total death: 166; 1.48 (0.62–1.66); CV events: 98; 1.38 (0.60–3.19)	1.67	Age, BMI, smoking, SHBG, cancer, diabetes	6

Nakashima et al. 2017 [23]	Japan	Prospective cohort	HD	902	63.4 ± 11.8	Lowest tertile 3 vs. highest	Total death: 123; 2.26 (1.21–4.23); CV events: 151; 1.19 (0.74–1.91); infectious events, 116; 2.12 (1.18–3.79)	2.06	Age, BMI, albumin, creatinine, CRP, SHBG, ACEI/ARB medication; diabetes, history of CVD	8

Yu et al. 2017 [24]	America	Retrospective cohort	HD and PD	624	58 ± 14	Lowest tertile 3 vs. highest	Total death: 108; 2.32 (1.33–4.06)	1.2	Age, race, diabetes; dialysis vintage, cause of ESRD, modality, dialysis access, CHF, CHD, albumin	7

Wu et al. 2018 [25]	Taiwan	Retrospective cohort	HD	137	71.7 ± 9.4	Low vs. high	Total death: 61; 3.39 (1.67–6.86); CV death: 36; 6.13 (2.27–16.53)	5.0	Age, BMI, body composition, SMMI, diabetes, hypertension, albumin, creatinine, hemoglobin, CRP	6

Unless specified, adjusted HR (95% CI) represents effect estimates of total testosterone. HR, hazard ratio; CI, confidence interval; HD, hemodialysis; PD, peritoneal dialysis; CKD, chronic kidney disease; CV, cardiovascular; BMI, body mass index; SMMI, skeletal muscle mass index; CRP, C-reactive protein; ACEI, angiotensin-converting enzyme inhibitors; ARB, angiotensin II receptor blocker; SHBG, sex hormone binding globulin; CVD, cardiovascular disease; CHF, congestive heart failure; ESRD, end-stage renal disease; CHD, coronary heart disease; FMD, flow-mediated dilation; eGFR, estimated glomerular filtration rate; CAD, coronary artery disease; and PWV, pulse wave velocity.

## Data Availability

All datasets generated for this study are included in this manuscript. Further information and requests can be directed to the corresponding author. In addition, the protocol of this meta-analysis is freely accessible at INPLASY (https://inplasy.com/wp-content/uploads/2022/05/INPLASY-Protocol-3342-1.pdf; registration number: INPLASY 202250085).

## References

[1] Mizdrak M., Kumrić M., Kurir T. T., Božić J. (2022). Emerging biomarkers for early detection of chronic kidney disease. *Journal of Personalized Medicine*.

[2] Brar A., Markell M. (2019). Impact of gender and gender disparities in patients with kidney disease. *Current Opinion in Nephrology and Hypertension*.

[3] Hill N. R., Fatoba S. T., Oke J. L. (2016). Global prevalence of chronic kidney disease - a systematic review and meta-analysis. *PLoS One*.

[4] Lima-Posada I., Bobadilla N. A. (2021). Understanding the opposite effects of sex hormones in mediating renal injury. *Nephrology*.

[5] Hu Z., Pei F., Zhou Z. (2017). Chronic kidney disease in Chinese postmenopausal women: a cross-sectional survey. *Nigerian Journal of Clinical Practice*.

[6] Bianchi V. E. (2018). Testosterone, myocardial function, and mortality. *Heart Failure Reviews*.

[7] Wang N., Wang L., Huang C. (2021). Association of total testosterone status with bone mineral density in adults aged 40-60 years. *Journal of Orthopaedic Surgery and Research*.

[8] Dandona P., Dhindsa S., Ghanim H., Saad F. (2021). Mechanisms underlying the metabolic actions of testosterone in humans: a narrative review. *Diabetes, Obesity and Metabolism*.

[9] Erenpreiss J., Fodina V., Pozarska R., Zubkova K., Dudorova A., Pozarskis A. (2020). Prevalence of testosterone deficiency among aging men with and without morbidities. *The Aging Male*.

[10] Mahmoud T., Borgi L. (2021). The interplay between nutrition, metabolic, and endocrine disorders in chronic kidney disease. *Seminars in Nephrology*.

[11] Valdivielso J. M., Jacobs-Cachá C., Soler M. J. (2019). Sex hormones and their influence on chronic kidney disease. *Current Opinion in Nephrology and Hypertension*.

[12] Dousdampanis P., Trigka K., Fourtounas C., Bargman J. M. (2014). Role of testosterone in the pathogenesis, progression, prognosis and comorbidity of men with chronic kidney disease. *Therapeutic Apheresis and Dialysis*.

[13] Garibotto G., Esposito P., Picciotto D., Verzola D. (2021). Testosterone disorders and male hypogonadism in kidney disease. *Seminars in Nephrology*.

[14] Page M. J., McKenzie J. E., Bossuyt P. M. (2021). The PRISMA 2020 statement: an updated guideline for reporting systematic reviews. *BMJ*.

[15] Stang A. (2010). Critical evaluation of the Newcastle-Ottawa scale for the assessment of the quality of nonrandomized studies in meta-analyses. *European Journal of Epidemiology*.

[16] Danesh J., Collins R., Appleby P., Peto R. (1998). Association of fibrinogen, C-reactive protein, albumin, or leukocyte count with coronary heart disease: meta-analyses of prospective studies. *JAMA*.

[17] Carrero J. J., Qureshi A. R., Parini P. (2009). Low serum testosterone increases mortality risk among male dialysis patients. *Journal of the American Society of Nephrology*.

[18] Gungor O., Kircelli F., Carrero J. J. (2010). Endogenous testosterone and mortality in male hemodialysis patients: is it the result of aging?. *Clinical Journal of the American Society of Nephrology*.

[19] Yilmaz M. I., Sonmez A., Qureshi A. R. (2011). Endogenous testosterone, endothelial dysfunction, and cardiovascular events in men with nondialysis chronic kidney disease. *Clinical Journal of the American Society of Nephrology*.

[20] Kyriazis J., Tzanakis I., Stylianou K. (2011). Low serum testosterone, arterial stiffness and mortality in male haemodialysis patients. *Nephrology Dialysis Transplantation*.

[21] Khurana K. K., Navaneethan S. D., Arrigain S., Schold J. D., Nally J. V., Shoskes D. A. (2014). Serum testosterone levels and mortality in men with CKD stages 3-4. *American Journal of Kidney Diseases*.

[22] Bello A. K., Stenvinkel P., Lin M. (2014). Serum testosterone levels and clinical outcomes in male hemodialysis patients. *American Journal of Kidney Diseases*.

[23] Nakashima A., Ohkido I., Yokoyama K., Mafune A., Urashima M., Yokoo T. (2017). Associations between low serum testosterone and all-cause mortality and infection-related hospitalization in male hemodialysis patients: a prospective cohort study. *Kidney International Reports*.

[24] Yu J., Ravel V. A., You A. S. (2017). Association between testosterone and mortality risk among U.S. Males receiving dialysis. *American Journal of Nephrology*.

[25] Wu H. C., Lee L. C., Wang W. J. (2018). The association between serum testosterone and mortality among elderly men on hemodialysis. *Journal of Clinical Laboratory Analysis*.

[26] van der Burgh A. C., Khan S. R., Neggers S., Hoorn E. J., Chaker L. (2022). *The Role of Serum Testosterone and Dehydroepiandrosterone Sulfate in Kidney Function and Clinical Outcomes in Chronic Kidney Disease: A Systematic Review and Meta-Analysis*.

[27] Marriott R. J., Harse J., Murray K., Yeap B. B. (2021). Systematic review and meta-analyses on associations of endogenous testosterone concentration with health outcomes in community-dwelling men. *BMJ Open*.

[28] Ruige J. B., Mahmoud A. M., De Bacquer D., Kaufman J. M. (2011). Endogenous testosterone and cardiovascular disease in healthy men: a meta-analysis. *Heart*.

[29] Corona G., Rastrelli G., Di Pasquale G., Sforza A., Mannucci E., Maggi M. (2018). Endogenous testosterone levels and cardiovascular risk: meta-analysis of observational studies. *The Journal of Sexual Medicine*.

[30] Xu L., Freeman G., Cowling B. J., Schooling C. M. (2013). Testosterone therapy and cardiovascular events among men: a systematic review and meta-analysis of placebo-controlled randomized trials. *BMC Medicine*.

[31] Bhasin S., Brito J. P., Cunningham G. R. (2018). Testosterone therapy in men with hypogonadism: an endocrine society clinical practice guideline. *Journal of Clinical Endocrinology & Metabolism*.

[32] Gagliano-Jucá T., Basaria S. (2019). Testosterone replacement therapy and cardiovascular risk. *Nature Reviews Cardiology*.

[33] Hudson J., Cruickshank M., Quinton R. (2022). Adverse cardiovascular events and mortality in men during testosterone treatment: an individual patient and aggregate data meta-analysis. *The Lancet Healthy Longevity*.

[34] Barone B., Napolitano L., Abate M. (2022). The role of testosterone in the elderly: what do we know?. *International Journal of Molecular Sciences*.

[35] Bhasin S. (2021). Testosterone replacement in aging men: an evidence-based patient-centric perspective. *The Journal of Clinical Investigation*.

[36] Li S. Y., Zhao Y. L., Yang Y. F. (2020). Metabolic effects of testosterone replacement therapy in patients with type 2 diabetes mellitus or metabolic syndrome: a meta-analysis. *The Internet Journal of Endocrinology*.

[37] Yeo J. K., Koo H. S., Yu J., Park M. G. (2020). Effects of testosterone treatment on quality of life in patients with chronic kidney disease. *American Journal of Men’s Health*.

[38] Edey M. M. (2017). Male sexual dysfunction and chronic kidney disease. *Frontiers of Medicine*.

[39] García-Cruz E., Carrión A., Ajami T. (2018). The patient’s comorbidity burden correlates with the erectile dysfunction severity. *Actas Urológicas Españolas*.

[40] Mihai S., Codrici E., Popescu I. D. (2018). Inflammation-related mechanisms in chronic kidney disease prediction, progression, and outcome. *J Immunol Res*.

